# Surgical Management of Severe Mandibular Actinomycosis: Segmental Mandibulectomy and Fibula Free Flap for Optimal Outcomes

**DOI:** 10.7759/cureus.52212

**Published:** 2024-01-13

**Authors:** Paula Maria Leite, Carolina F Chaves, Bruno Morgado, Horácio Zenha, Horácio Costa

**Affiliations:** 1 Plastic and Reconstructive Surgery, Centro Hospitalar de Vila Nova de Gaia/Espinho, Vila Nova de Gaia, PRT; 2 Microsurgery and Experimental Surgery Unit, University of Aveiro, Aveiro, PRT; 3 Faculty of Medicine and Biomedical Sciences, University of Algarve, Faro, PRT

**Keywords:** mandible, free flap reconstruction, fibular free flap, actinomycosis, actinomyces

## Abstract

Actinomycosis is a chronic, suppurative, granulomatous bacterial infection primarily associated with *Actinomyces israelii*. The condition can be categorized into three distinct clinical types based on the affected anatomical region: cervicofacial, pulmonary, or abdominopelvic actinomycosis. The standard treatment for actinomycosis involves antibiotic therapy, with an empiric penicillin regimen as the first-line approach. Surgical interventions comprise curettage of the affected bone, resection of necrotic tissues, excision of existing sinus tracts, and drainage of abscesses. These procedures are considered a last resort for cases of actinomycosis unresponsive to antibiotic therapy. In this context, we present a case of severely unresponsive actinomycosis that necessitated aggressive surgical resection of the infected mandibular bone, followed by immediate reconstruction using a fibula-free flap. The outcome yielded both favorable functional and aesthetic results.

## Introduction

*Actinomyces *species (spp.) are Gram-positive filamentous bacilli frequently found in the human commensal flora, specifically in the oropharynx, gastrointestinal tract, and urogenital tracts [1-7]. Under normal conditions, *Actinomyces* has low pathogenicity levels, as it is unable to infiltrate healthy tissue [1,2,7]. However, in rare cases, under predisposing conditions, such as an immunocompromised state, decreased tissue oxygenation, or tissue injury, these bacteria might lead to an infection known as actinomycosis [1,2,5,7].

Actinomycosis can be characterized as a chronic, suppurative, granulomatous bacterial infection, most commonly caused by *Actinomyces israelii*, and less frequently by *Actinomyces gerencseriae* [1,3,4,6,7].

Actinomycosis can be categorized into three distinct clinical types based on the affected area: cervicofacial, pulmonary, or abdominopelvic actinomycosis. Notably, cervicofacial actinomycosis stands as the most prevalent type [1,3,4,6].

The standard treatment for actinomycosis involves antibiotic therapy, with an empiric penicillin course as the first-line approach [1-5]. Depending on the clinical stage of the disease, additional surgical interventions may be necessary. These may encompass curettage of the affected bone, resection of necrotic tissues, excision of existing sinus tracts, and drainage of abscesses [2,6,7].

In this article, we present a case of cervicofacial actinomycosis that exhibited significant resistance to prolonged periods of antibiotherapy and multiple surgical interventions involving washing and curettage. Consequently, the decision was made to escalate the treatment to encompass extensive resection and reconstruction using a free flap. This approach aimed to achieve a curative outcome, as elaborated upon in the subsequent sections.

## Case presentation

A 60-year-old woman presented with a five-month history of pain and swelling in the right submandibular area. The patient underwent three brief antibiotic cycles during this period, including amoxicillin, metronidazole, and, most recently, piperacillin/tazobactam. While there was temporary relief of pain, there were no sustained long-term improvements.

Extra-orally, a slight facial asymmetry was noted, attributed to swelling in the right submandibular region that was tender on palpation and accompanied by drainage through an oral cutaneous fistula. In the intra-oral examination, necrotic bone was observed on the right side of the mandibular body, specifically in the molar region. Oral hygiene was deemed acceptable, with no evidence of active caries or other dental or periodontal diseases. During the anamnesis, the patient disclosed a weekly regimen of alendronic acid for osteoporosis, initiated eight years prior. There was no reported history of recent dental procedures or trauma.

Considering the clinical observation of exposed necrotic bone in the mandible and the patient's history of long-term bisphosphonate therapy, medication-related osteonecrosis of the jaw (MRONJ) was suspected. A biopsy of the lesion was conducted, confirming this diagnosis. In the histological examination, findings consistent with colonies of *Actinomyces* were identified, leading to the additional diagnosis of mandibular actinomycosis. Unfortunately, the isolation of *Actinomyces* in culture was not feasible.

In an attempt to concurrently address both MRONJ and mandibular actinomycosis, in addition to immediately stopping the weekly regimen of alendronic acid, a treatment protocol involving systemic antibiotics and surgical curettage was initiated. The patient underwent an initial one-month cycle of ceftriaxone, followed by a 24-month course of amoxicillin, coupled with multiple surgical interventions for washing and curettage of the necrotic bone. Following this treatment period, a maxillofacial computed tomography (CT) scan was conducted, revealing the progression of mandibular osteonecrosis in comparison to previous examinations (Figure 1).

**Figure 1:** Preoperative CT bone window (A and B) Osteomyelitis of the right mandibular body with bone sequestration (white arrow). (C) Sinus tract in the right submandibular region (white arrow) and cellulitis in the right submandibular area.

At this juncture, despite an extended period of over two years of antibiotic therapy and multiple interventions involving washing and curettage of the affected bone, the infection remained uncontrolled, and the patient exhibited both clinical and radiological deterioration. Subsequently, a consensus was reached that a more invasive treatment strategy was necessary. The proposed approach entailed the resection of the infected mandibular bone followed by immediate reconstruction using a fibula-free flap. The patient provided consent for the procedure, and a right segmental mandibulectomy was performed, resulting in a class II bone defect as per the Zenha H et al. classification [8]. Simultaneously, fistulectomy of the submandibular cutaneous fistula was carried out using a submandibular approach (Figure 2).

**Figure 2:** Right submandibular sinus tract with pre-operative excision marking

A bone segment from the left fibula was harvested by following the pre-established 3D cutting guides [9]. No skin paddle was included. The fibula was fixated to the remaining mandible by a pre-molded plate (Figure 3).

**Figure 3:** Reconstruction with a fibula-free flap (A) 3D cutting guides in the osteo-muscular left fibula; (B) Fibula flap harvesting; (C) Fixation of the remaining mandible through osteosynthesis using a pre-molded plate

End-to-end microvascular anastomoses were performed connecting the peroneal artery and concomitant vein to the right facial artery and vein in the cervical region. The postoperative period was uneventful. The anatomopathological examination of the surgical specimen unveiled osteonecrosis and acute osteitis lesions. At the one-year follow-up, the osseointegration of the vascularized fibula was assessed using a maxillofacial CT scan, revealing robust osseointegration without signs of osteomyelitis, osteonecrosis, or alterations in soft tissues (Figure 4).

**Figure 4:** One-year post-surgery CT scan (A, B, and C) Axial CT bone window illustrating robust osseointegration of the fibula-free flap. (D, E, and F) CT bone window with 3D reconstruction

The aesthetic and functional outcomes were excellent (Figure 5), with the patient reporting no functional limitations and expressing high levels of aesthetic satisfaction.

**Figure 5:** Postoperative results at one year (A) Left fibula donor site with a linear scar; (B) Frontal facial view, showing no asymmetry; (C) Right profile view demonstrating a well-defined mandible contour

## Discussion

As previously mentioned, *Actinomyces* are typically unable to infiltrate healthy tissue, requiring underlying conditions for infection to occur [1,2,5,7]. Concerning cervicofacial actinomycosis, the predisposing condition is often unclear; however, common risk factors for this disease include an immunocompromised state, chronic infections, and breaches of the oral mucosa [1-3,5,6]. In this instance, the most probable cause was the disruption of the oral mucosa due to the evolving MRONJ.

The clinical manifestations of actinomycosis are nonspecific, resembling symptoms of various infectious, inflammatory, or even malignant diseases, contributing to frequent misdiagnoses [1,2,5]. The predominant clinical feature in cervicofacial actinomycosis is facial swelling, often accompanied by pain and induration [1,5-7]. Following its initiation, the infection can extend to adjacent tissues without respect for anatomical barriers, resulting in the common occurrence of sinus tracts with suppurative drainage [1,2,4,5]. While not pathognomonic, the presence of sulfur granules, characterized by yellow grains with an intense foul smell, is observed in 40% of cases and should strongly indicate the likelihood of actinomycosis [1,3-7]. Nevertheless, it is important to highlight that this distinctive feature was absent in our patient.

A classification system proposed by Karanfilian KM, et al. for cervicofacial actinomycosis categorizes the disease into three stages based on its clinical features [1]. Stage one is characterized by the initial swelling of the perimandibular soft tissues. Stage two involves the progressive spread into adjacent tissues over time, accompanied by induration of the affected area and the formation of sinus tracts containing purulent material, which may include sulfur granules. Stage three represents the final stage and involves a generalized infection with invasion of the cranium or the bloodstream [1]. According to the clinical features, this patient is classified as having stage two cervicofacial actinomycosis.

The diagnosis is established through the culture and isolation of the bacteria, preferably from a tissue sample. Nevertheless, in most cases, isolation of *Actinomyces* is not feasible due to challenging growth conditions and the frequent administration of prior antibiotic therapy [1-3,6,7]. Histological examination can provide additional support for the diagnosis of actinomycosis [1-4,6,7]. Initial hematological studies and imaging techniques, such as CT scans and magnetic resonance imaging, typically yield nonspecific findings [1,2]. In this instance, the diagnosis was established through histological examination, revealing findings consistent with the presence of *Actinomyces* colonies.

The conventional approach for treating actinomycosis involves antibiotic therapy. *Actinomyces* spp. exhibit heightened sensitivity to beta-lactams; consequently, the initial course of treatment typically involves empiric penicillin [1-5]. The duration of treatment exhibits considerable variability, ranging from a few weeks to more than a year. When coupled with surgical intervention, the duration of antibiotic therapy tends to be shorter [1-3,6,7]. Surgical modalities encompass curettage of the affected bone, resection of necrotic tissues, excision of sinus tracts, and drainage of abscesses. These interventions may serve as a final recourse for cases of actinomycosis resistant to antibiotic therapy, aiming to disrupt and eliminate the fibrous tissue surrounding the affected region, which may impede antibiotic penetration [2,6,7]. In this particular instance, we encountered a case of markedly unresponsive actinomycosis, wherein the infection persisted despite more than two years of appropriate antibiotic therapy and multiple surgical interventions involving curettage of the affected bone. In response to the continued progression of the infection, a more aggressive approach was undertaken, involving the resection of the infected mandibular bone and immediate reconstruction. For the reconstruction, a free, vascularized osteo-muscular fibula flap was chosen.

The benefit inherent in the free tissue transfer concept lies in its vascularization. Free vascularized bone flaps have demonstrated faster healing and greater reliability, especially in instances involving contamination of the recipient site wound [10]. Additionally, these flaps possess a clearly defined vascular supply, enabling multiple osteotomies, a particularly crucial aspect in craniofacial contouring procedures, as well as allowing future oral rehabilitation with implants [10-12].

Concerning the donor site, there was acceptable morbidity, a common occurrence with this flap. This manifested as a linear scar and minimal functional disability, primarily involving some discomfort in ankle function and range of movement during more strenuous physical exertion [10,11].

## Conclusions

Actinomycosis is an uncommon condition, with cervicofacial involvement being its most prevalent manifestation. The difficulty in diagnosing this infection arises from its nonspecific symptoms and imaging findings. Given its capacity to propagate to surrounding tissues without regard for anatomical barriers, this infection can pose a life-threatening risk, underscoring the critical importance of early diagnosis and appropriate treatment. Typically, treatment involves prolonged courses of antibiotics, primarily penicillin, alongside concurrent surgical interventions. In instances where there is an inadequate response to appropriate antibiotic regimens and surgical curettage, more aggressive strategies become necessary, involving extensive soft tissue and bone resections, as well as free vascularized tissue transfers to the head and neck region.
